# LINC01315 Impairs microRNA-211-Dependent DLG3 Downregulation to Inhibit the Development of Oral Squamous Cell Carcinoma

**DOI:** 10.3389/fonc.2020.556084

**Published:** 2020-09-28

**Authors:** Fu-Bo Chen, Peng Wu, Rong Zhou, Qi-Xiang Yang, Xu Zhang, Rao-Rao Wang, Sheng-Cai Qi, Xi Yang

**Affiliations:** ^1^Department of Stomatology, Shanghai Tenth People’s Hospital, Tongji University School of Medicine, Shanghai, China; ^2^Department of Othorpaedics, Shanghai Tenth People’s Hospital, Tongji University School of Medicine, Shanghai, China; ^3^Department of Oral & Maxillofacial - Head & Neck Oncology, Ninth People’s Hospital, Shanghai Jiao Tong University School of Medicine, Shanghai, China

**Keywords:** oral squamous cell carcinoma, LINC01315, microRNA-211, DLG3, Hippo signaling pathway, proliferation, migration, invasion

## Abstract

Recent studies have revealed that long non-coding RNAs (lncRNAs) involve in the progression of oral squamous cell carcinoma (OSCC). These lncRNAs have emerged as biomarkers or therapeutic targets for OSCC. We here aimed to investigate the role of lncRNA LINC01315 in OSCC and the related mechanisms. LINC01315 and DLG3 were determined to be poorly expressed while microRNA-211 (miR-211) was highly expressed in OSCC tissues and cells using RT-qPCR and western blot analysis. Based on the results obtained from dual-luciferase reporter gene, RIP, and FISH assays, LINC01315 was found to upregulate DLG3 expression by competitively binding to miR-211. Upon altering the expression of LINC01315, and/or miR-211 in OSCC cells with shRNA, mimic, or an inhibitor, we assessed their effects on OSCC cell proliferation, migration, invasion, and apoptosis. LINC01315 knockdown enhanced OSCC cell proliferation, migration and invasion, but dampened their apoptosis, all of which could be reversed by miR-211 inhibition. Elevation of DLG3, a target gene of miR-211, activated the Hippo signaling pathway, whereby suppressing OSCC progression *in vitro*. Finally, their roles in tumor growth were validated *in vivo*. These findings suggest that LINC01315 elevates DLG3 expression by competitively binding to miR-211, thereby suppressing OSCC progression.

## Introduction

Oral squamous cell carcinoma (OSCC) is one of the most commonly occurring malignancies around the world (1). It has been shown that alcohol and tobacco abuse, as well as human papilloma virus infection are the major risk factors of OSCC (2). The mortality and morbidity of OSCC remain quite high, despite the existence of treatments such as surgery and radiotherapy (3). Hence, it is imperative to achieve a better understanding of the pathogenic mechanisms of OSCC to facilitate the discovery of more effective therapeutic targets (4). In recent years, researchers has revealed that certain RNAs, such as long non-coding RNA (lncRNA) LINC01315 and microRNA-211 (miR-211) are critical for the development of OSCC (5, 6).

LncRNAs, a type of RNA transcript with more than 200 nucleotides, are transcribed from certain loci in the mammalian genome that is involved in regulation of gene expression and other cellular processes (7). In primary tumors and metastases, lncRNAs exhibit differential expression patterns (8). Furthermore, results obtained from a previous study have confirmed the abnormal expression of LINC01315 in OSCC (6). Moreover, a competing endogenous relationship between lncRNAs and miRNAs has been recently identified (9), which might be implicated in tumorigenesis. Indeed, miRNAs exert crucial roles in the development of human diseases, particularly in cancer, and they can act as tumor suppressors or oncogenes in various cancers, which have made them to be attractive biomarkers and novel therapeutic targets (10). Previous research has emphasized the crucial tissue-specific role of miR-211 in carcinogenesis (11). Indeed, Chen et al. have revealed that miR-211 plays an oncogenic role in OSCC and that its expression is a predictor of poor OSCC prognosis (12). Additionally, miRNAs can modulate gene expression post-transcriptionally by interacting with the 3′-UTR of specific target mRNAs (13). miR-211 is presumed to contain complementary sequences for disks large homolog 3 (DLG3) and LINC01315, according to prior predicted results of lncRNA-miRNA interactions and miRNA-mRNA interactions. Hence, we speculated that the interactions among LINC01315, miR-211 and DLG3 might participate in the progression of OSCC.

DLG3 regulates the NMDA receptor signaling pathway in neurons, which results in synaptic plasticity (14). Recently, DLG3 exhibits low expression in several cancers, including colon cancer, glioblastoma and lung cancer (15). A recent study has demonstrated that up-regulated DLG3 activated the Hippo signaling pathway, thereby suppressing breast cancer cell proliferation and promoting their apoptosis (16). The Hippo signaling pathway plays a crucial role in tissue development and homeostasis, acting in multiple cancer types *via* its core components, which include mammalian sterile 20-like 1/2 (MST1/2), large tumor suppressor 1/2 (LATS1/2), and Yes kinase-associated protein (YAP) (17). Suppression of the Hippo signaling pathway potentially confers chemoresistance to OSCC cells (18). A transcriptional co-activator with PDZ-binding motif, TAZ, which is a downstream effector of the Hippo signaling pathway, can induce epithelial-to-mesenchymal transition in OSCC (19). In addition, a recent work has suggested that lncRNA LEF1-AS1 promotes the progression of OSCC *via* upregulating YAP and blocking the Hippo signaling pathway (20). Based on the findings above, we hypothesized that LINC01315 may regulate the progression of OSCC by mediating miR-211, DLG3 and the Hippo signaling pathway. To test this hypothesis, we recruited OSCC patients for tissue donation, and investigated the clinical significance of LINC01315 and its potential downstream mechanisms regarding miR-211, DLG3 and Hippo signaling pathway in tumor specimens. Moreover, we analyzed the effects of these molecules on the biological functions of OSCC cells both *in vitro* and *in vivo*.

## Methods

### Study Subjects

OSCC tissues were collected from 94 patients who received surgical treatment at the Ninth People’s Hospital, Shanghai Jiao Tong University School of Medicine from January 2015 to March 2016. After surgeries, tissue samples were immediately collected and stored at −80°C. Adjacent normal tissues were collected at 0.5 cm away from the OSCC tumor margins. All patients enrolled in the experiment had given signed informed consent and the project was approved by the Ethics Committee of Ninth People’s Hospital, Shanghai Jiao Tong University School of Medicine.

### Cell Culture

Five commonly used OSCC cell lines (SAS, SCC25, HN4, HN6 and CAL-27), and NHOK (Cell Bank of Chinese Academy of Sciences, Shanghai, China) were selected for this experiment. After resuscitation, the cells were then cultured in Dulbecco’s modified Eagle’s medium (DMEM) (Gibco, Grand Island, NY, United States) supplemented with 10% fetal bovine serum (FBS), and incubated at 37°C in a saturated humidity incubator (Thermo Fisher Scientific Inc., Waltham, MA, United States) with 5% CO_2_. At 80% confluence, the cells were detached with 0.25% trypsin and sub-cultured at the ratio of 1:3.

### *In silico* Analysis

The gene expression profiles related to OSCC (GSE30784, GSE74530 and GSE45238) and the annotation files were retrieved from the Gene Expression Omnibus (GEO) database^1^ (last accessed date: November 13, 2018) for systematic analysis of differential expression of genes, lncRNAs and miRNAs in OSCC. The “limma” package of R language was applied for differentiation analysis between the OSCC samples and control samples with | logFoldChange| > 2 and *p* value <0.05 as the screening standards for differentially expressed genes. At the same time, the R language “pheatmap” package was used to construct the heatmap for visualizing differential gene expression. The lncRNA-binding miRNA was predicted using the RNA22 website^2^ (last accessed date: November 13, 2018), while the potential target genes of miR-211 were predicted by the microRNA.org website^3^ (last accessed date: December 23, 2018), followed by retrieval of differential expression in the microarray dataset.

### Lentivirus Packaging and Construction of Cell Lines

The gene sequences of LINC01315 and DLG3 were found in the National Center for Biotechnology Information (NCBI) database available at https://www.ncbi.nlm.nih.gov/ (last accessed date: December 26, 2018). The short hairpin RNA (shRNA) against LINC01315 (sh-LINC01315) sequence was supplied by Addgene Company (Cambridge, MA, United States), and the shRNA against DLG3 (sh-DLG3) sequence by Sigma-Aldrich (St. Louis, MO, United States). The two shRNAs were inserted separately into the PLKO.1-Puro (Sigma-Aldrich) carrier. After confirmatory sequencing, the above plasmids were independently co-transfected with psPAX2 and pMD2.G (Addgene, Cambridge, MA, United States) into 293T cells. Then, the infected SAS and HN4 cells were cultured with puromycin (Sigma-Aldrich) for selection of stable cell lines, which were designated as SAS/HN4-sh-DLG3 or SAS/HN4-sh-LINC01315.

### Cell Transfection

Cells were seeded in six-well plates with 10^5^ cells in each well. When cell confluence reached 80%, transfection was performed on pcDNA3.1-miR-211 using the Lipofectamine 2000 reagents (Invitrogen, Carlsbad, CA, United States). Serum-free DMEM (250 μL; Gibco, Carlsbad, CA, United States) was used to dilute 4 μg of the target plasmid and 10 μL of Lipofectamine 2000, respectively, both of which were allowed to stand for 5 min. The diluted plasmids and the Lipofectamine 2000 were mixed and allowed to stand for 20 min before addition to the culture wells, which were incubated in a 5% CO_2_ incubator at 37°C. After incubation for 6 h, the medium was renewed with complete medium and the cells were collected after another 48 h of incubation.

### Immunohistochemistry

OSCC tissues were fixed in 10% formaldehyde for 24 h, paraffin-embedded and sliced into sections. The sections were then deparaffinized in methylbenzene, and dehydrated using a graded ethanol series (100% I, 100% II, 95%, 85% and 75%, for 3 min each). The sections were then incubated with antigen retrieval fluid at 97°C for 5 min and immersed in 3% deionized water containing H_2_O_2_ for 20 min. After that, the sections were exposed to normal goat serum for 15 min, followed by incubation with rabbit anti-mouse DLG3 (1:100, ab3438, Abcam Inc., Cambridge, United Kingdom) at 4°C overnight. Then, the sections were incubated with goat anti-rabbit immunoglobulin G (IgG) (1:100, ab205718, Abcam Inc.) at room temperature for 30 min and with streptavidin-labeled horseradish peroxidase (HRP) at room temperature for 30 min. The sections were subsequently stained with diaminobenzidine and counter-stained with hematoxylin, followed by microscopic observation (Nikon, Tokyo, Japan).

### Subcellular Location of LINC01315

Bioinformatics tools^4^ (last accessed date: November 13, 2018) were used to obtain information about the subcellular localization of LINC01315. Then, as described previously (21), we used the fluorescent *in situ* hybridization (FISH) for verification, following the instructions provided in the Ribo^TM^ lncRNA FISH Probe Mix (Red) kit (Guangzhou RiboBio Co., Ltd., Guangzhou, China). SAS cells were seeded in a six-well plate for 1 day to attain cell confluence of about 80%. On the next day, the cells were fixed with 4% paraformaldehyde (1 mL) at room temperature, followed by treatment with proteinase K (2 μg/mL), glycine, and acetylation. The cells were then incubated with 250 μL of pre-hybridization solution at 42°C for 1 h and subsequently incubated with 250 μL of 300 ng/mL hybridization solution containing the probes overnight at 42°C. On the next day, the cells were stained for 5 min in a 24-well plate with Hoechst solution diluted in phosphate buffered saline tween-20 at the ratio of 1:800. Before observation, cells were mounted in anti-fluorescence quencher. Five different randomly selected fields were observed and photographed under the fluorescence microscope (Olympus, Tokyo, Japan).

### RNA Immunoprecipitation (RIP) Assay

Cells were lysed using lysis buffer (25 mM Tris-HCl, pH = 7.4; 150 mM NaCl; 0.5% Non-idet P-40; 2 mM ethylenediaminetetraacetic acid; 1 mM NaF, and 0.5 mM dithiothreotol) containing RNasin (Takara, Tokyo, Japan) and protease inhibitor (P1005, Beyotime Biotechnology Co., Shanghai, China). Next, the lysate was centrifuged at 12,000 × *g* for 200 min and the supernatant was collected, followed by the addition of anti-Ago-2 magnetic beads. Lysate added with anti-IgG as control. After incubation at 4°C for 4 h, the magnetic beads were washed with washing buffer (50 mM Tris-HCl; 300 mM NaCl, pH = 7.4; 1 mM MgCl 2; 0.1% Non-idet P-40) and RNA was extracted from the magnetic beads using TRIzol reagents for reverse transcription-quantitative polymerase chain reaction (RT-qPCR).

### Immunofluorescence

The cells were fixed with 4% paraformaldehyde at room temperature for 15 min, followed by incubation with 0.1% Triton X-100 at room temperature for 20 min. After that, the samples were blocked for 30 min in 10% rabbit serum and incubated with primary rabbit anti-human antibody to YAP (1:100, ab52771, Abcam Inc.) at 4°C overnight, followed by incubation with TRICT-labeled goat anti-rabbit antibody against IgG (1:100, ab205718, Abcam Inc.). Then, cell nuclei were visualized with 4’6-diamidino-2-phenylindole (5 μg/mL) for 2 min and mounted with anti-fluorescence quencher, which were then observed under the fluorescence microscope.

### Dual-Luciferase Reporter Assay

Initially, binding site between miR-211 and DLG3 or between miR-211 and LINC01315 was predicted by RNA22 database (last accessed date: November 13, 2018) and microRNA.org database (last accessed date: December 23, 2018). The binding site between miR-211 and LINC01315, as well as the binding site between miR-211 and DLG3 were directly mutated. The sequences namely LINC01315-wild type (WT) and LINC01315-mutant type (MUT), DLG3-WT-3′-untranslated region (3′-UTR) and DLG3-MUT-3′-UTR (Shanghai Genechem Co., Ltd., Shanghai, China) were separately ligated to pisCHECK2 vector (Ambion, Austin, TX, United States) (Table 1). After sequence verification, LINC01315-WT and LINC01315-MUT, and DLG3-WT-3′-UTR, and DLG3-MUT-3′-UTR plasmids were transfected respectively with miR-211 mimic negative control (NC) and miR-211 mimic into the SAS cell line. Luciferase activity detection was carried out using the dual-luciferase reporter gene assay kit (Promega, Madison, WI, United States). The cell lysate (20 μL) was incubated with 100 μL of LARII solution, which was mixed and placed in a luminescent detector (GloMax 2020, Promega, Madison, WI, United States) to detect its firefly luminance. After applying the Stop & Glo detection solution to stop the reaction, the renilla luminance was measured as the internal reference, and the ratio of firefly luminance/renilla luminance was calculated.

**TABLE 1:** Sequences for dual-luciferase reporter gene assay.

**Target**	**Sequences**
LINC01315-WT	3′-GAGGGAAAGAGACCGGGAGUC-5′
LINC01315-MUT	3′-TGTTTCCCGGTACCTTGCTTC-5′
has-miR-211	3′-CGCUUCCUACUGUUUCCCUU-5′
DLG3-WT-3′-UTR	3′-UAGGGAAAAACGGAAGUUCG-5′
DLG3-MUT-3′-UTR	3′-UGATTGCCAGCTTGGATUCG-5′

*WT, wild type; MUT, mutant type; 3′-UTR, 3′-untranslated region.*

### 3-(4,5-Dimethylthiazol-2-yl)-2, 5-Diphenyltetrazolium Bromide (MTT) Assay

Cells in the logarithmic phase were harvested, 200 μL of which were seeded in each well of a 96-well plate after adjusting the cell density to 3 × 10^4^ cells/mL (the marginal well was filled with sterile PBS). Each group that contained different transfection plasmids had six duplicated wells, with five plates in total. The adherence of cells was observed after 12 h incubation. In addition, each well was unceasingly incubated for 1, 2, 3, 4, and 5 days, and after each time point, cells were further incubated with the addition of 20 μL of MTT (Hyclone, South Logan, UT, United States) for 4 h, followed by mixing with 100 μL of dimethyl sulfoxide (Sigma-Aldrich) with shaking for 1 min. The absorbance of OD490 was measured with a microplate reader.

### Scratch Test

The cells in the logarithmic phase were harvested and seeded in a six-well plate at a density of 10^6^ cells/well. A marker pen was used to draw a line on the back of plate uniformly as a registration point for taking photomicrographs. After the cells had attained confluence on the surface of the six-well plate, the primary culture solution was replaced with 1% FBS to starve the cells for 12 h. Using a straight ruler as a guide, a 200-μL pipette tip was applied to create a vertical scratch on the bottom of the six-well plate. Photomicrographs were taken at 0 and 24 h to record the cell migration. Scratch width was calculated as follows: a total of 15 evenly spaced lines were drawn on each of the scratched picture and the width across the 15 lines was measured to obtain the average width of the scratch. Cell migration rate (%) = (1 - scratch width/initial scratch width) × 100%.

### Transwell Assay

The Matrigel (354234, BD Biosciences San Jose, CA, United States) was mixed with serum-free cell culture medium at the ratio of 1:1 and polymerized into a gel at 37°C in a Transwell chamber (Corning, NY, United States) in a volume of 50 μL/well. Cells at the logarithmic phase were starved for 24 h with 1% FBS. After detachment, the cells were resuspended in serum-free medium to prepare cell suspension (10^6^ cells/mL), and 50 μL portions were mixed with 50 μL of 2% FBS prior to transferring to the corresponding Transwell chambers. The cell culture medium (600 μL) containing 10% FBS was added to the lower layer of the chamber. The cells were cultured at 37°C in an incubator with 5% CO_2_, saturated humidity and rich oxygen for 24 h. On the next day, the cells were removed from Transwell chamber and fixed with 4% paraformaldehyde, followed by crystal violet staining. Five fields with fixed positions were randomly selected by the five-point sampling method to count cells under an inverted microscope at high magnification (400×).

### Western Blot Analysis

Radioimmunoprecipitation assay (RIPA) lysis buffer (P0013C, Beyotime) was used to lyse tissues and cells. The lysates of tissues and cells were centrifuged at 14,000 rpm and 4°C to collect total protein, cytoplasmic protein and nuclear protein in the supernatant, which were stored at −80°C until use. The extracted protein concentration was measured by the bicinchonininc acid method (23225, Pierce, Rockford, IL, United States). Then, 50 μg protein was collected and dissolved in 2 × SDS loading buffer solution and boiled for 5 min. Next, the protein samples were subjected to electrophoretic separation using 4% stacking gel and 10% stacking gel. Separated proteins were transferred onto a membrane, which was subsequently mounted with 0.5% bovine serum albumin. The membrane was incubated overnight with rabbit anti-human antibodies (Abcam Inc.) against DLG3 (1:1000, ab3438), MST2 (1:1000, ab70546), MST1 (1:1000, ab124787), LATS1 (1:1000, ab70561), YAP (1:1000, ab52771) and glyceraldehyde-3-phosphate dehydrogenase (GAPDH) (1:1000, ab70699). The next day, after washing in buffer, the proteins were incubated with HRP-labeled goat anti-rabbit antibody against IgG (1:1000, ab205718, Abcam Inc.) at room temperature for 2 h. The enhanced chemiluminescence (32109, Invitrogen) was used for color development. The images were captured using Bio-rad microscopy imaging system and gray value of protein bands were analyzed using Image Lab.

### RNA Isolation and Quantitation

Total RNA was extracted with the TRIzol reagent (15596-026, Invitrogen) and the concentration of the extracted RNA was measured with a spectrophotometer. Total RNA was reversely transcribed into complementary DNA (cDNA) using the oligodT method, and real time qPCR was performed using the SYBRgreen reagent. The primer sequences of DLG3 were as follows: (forward) 5′-AAAGTGAGCAGATCGGTGTGA-3′ and (reverse) 5′-CCTGTTAGACTCAATCATCCCCG-3′. The primer sequences of miR-211 were as follows: (forward) 5′-GGGAGTGGACCGGTACAA-3′ and (reverse) 5′-CAGTGCGTGTCGTGGAGT-3′. The primer sequences of LINC01315 were as follows: (forward) 5′- CGCCATCGATGTTATCGCAA-3′ and (reverse) 5′-GGCATCCACTTCATCGCTCA-3′. All primer sequences were designed and synthesized by Beijing Genomics Institute (BGI, Beijing, China). The reliability of the PCR results was evaluated by examining the disassociation curve. The relative quantification method (2^–Δ^ ^Δ^ ^*Ct*^ method) was adopted to calculate the relative expression of each target gene.

### Flow Cytometry

After 48 h of transfection, OSCC cells were collected in a flow tube, and centrifuged at 179 × *g* for 5 min, with the supernatant discarded. Then, the cells were recentrifuged and the supernatant again discarded. As per the instructions in the Annexin-V-fluorescein isothiocyante (FITC) apoptosis assay kit (Sigma-Aldrich), the cells were incubated with 150 μL of binding buffer and 5 μL of Annexin-V-FITC by shaking in the dark for 15 min at room temperature. Each tube was mixed with 100 μL of binding buffer and 5 μL of propidium iodide (PI) staining solution (Sigma-Aldrich). Apoptosis was subsequently determined by a flow cytometer (FACSCanto II, BD Biosciences, Franklin Lakes, NJ, United States).

### Xenograft Tumor in Nude Mice

A total of 36 specific pathogen-free male nude mice (weighing 14–16 g, aged 4 weeks, Shanghai SLAC Laboratory Animal Co., Ltd., Shanghai, China) were randomly assigned to six groups with six mice per group: sh-NC + inhibitor NC, sh-LINC01315 + inhibitor NC, sh-LINC01315 + miR-211 inhibitor, sh-DLG3 + inhibitor NC, sh-DLG3 + miR-211 inhibitor, and sh-NC + miR-211 inhibitor groups. SAS cells were resuspended in serum-free DMEM (Gibco) to prepare 1 × 10^7^ cells/mL cell suspensions and construct stable cell lines. The mice were anesthetized with ether, followed by routine disinfection and subcutaneous injection in backside with 100 μL cell suspension. The volume of the xenograft tumor was measured every 5 days and calculated in mm^3^ as: *V* = *A*^2^ × *B*/2 (where *A* indicates the long diameter, and *B* indicates the short diameter). The nude mice were euthanized after 35 days, whereupon the tumors were collected and weighed. These experimental animals were used exclusively for medical research and all operations were in accordance with the Guide for the Care and Use of Laboratory Animal by International Committees and approved by Animal Committee of Ninth People’s Hospital, Shanghai Jiao Tong University School of Medicine.

### Statistical Analysis

SPSS 21.0 (IBM Corp, Armonk, NY, United States) software was used for statistical analysis, and the mean value and standard deviations were calculated. Each experiment was conducted at least three times independently. Paired *t*-test was used to analyze the data between adjacent normal and cancer tissues, while unpaired *t*-test was used for the other two-group comparisons. One-way analysis of variance (ANOVA) was used for multi-group data analysis, followed by a Tukey’s multiple comparisons post-test. The repeated measures ANOVA was applied for the comparison of tumor volume at different time points. Correlations between LINC01315, miR-211 and DLG3 expression in the cancer tissues were analyzed by Pearson’s correlation coefficient. *p* < 0.05 was considered significantly different.

## Results

### LINC01315/miR-211/DLG3 Is Involved in the Progression of OSCC

In recent years, a growing number of studies have demonstrated the involvement of lncRNAs in OSCC. A lncRNA profile study has characterized the dysregulation of several lncRNAs in OSCC tissues, showing their predictive values for clinical stage and prognosis (22). Furthermore, lncRNAs have been linked to metastasis of OSCC in recent decades. For instance, lncRNA AC132217.4 can promote the metastasis of OSCC by upregulating the expression of IGF2 (23). LncRNA-p23154 has the potential to facilitate the invasion and metastasis of OSCC by regulating GLUT1-mediated glycolysis (24). These studies aroused our interest to perform *in silico* analyses of lncRNAs in OSCC samples.

Through differential analysis of the OSCC-related expression dataset GSE30784, we obtained 420 genes that were significantly over- or under-expressed in OSCC samples, among which LINC01315 was considerably downregulated in OSCC (Figure 1A). This was consistent with previous findings demonstrating the key significance of LINC01315 in oral carcinogenesis (6). Hence, LINC01315 was considered as the study subject of our OSCC research. Another independent OSCC-related expression dataset GSE74530 was retrieved from the GEO database, which concurred in showing downregulation of LINC01315 in OSCC (Figure 1B). For exploration purposes, the downstream regulatory mechanism of LINC01315 was further predicted. Subsequently, 85 differentially expressed miRNAs were retrieved from the OSCC-related miRNA expression dataset GSE45238 available on the GEO database (Figure 1C). The RNA22 database was used to predict the downstream miRNAs of LINC01315; the upregulated miRNAs in the expression dataset GSE45238 and the prediction results from the RNA22 database were then intersected, finally obtaining five miRNAs (Figure 1D), among which miR-211 expression exhibited the largest significant difference between OSCC tissues and adjacent normal tissues (Figure 1E). Hence, we selected miR-211 for particular examination. We then predicted a binding site between miR-211 and DLG3 from scrutiny of the database available on microRNA.org. Also, DLG3 was downregulated in samples from the OSCC expression dataset GSE30784 (Figure 1A). Therefore, we inferred that miR-211 might function in OSCC through interactions with DLG3, and LINC01315 might mediate miR-211 to regulate the expression of DLG3, thus influencing the development of OSCC.

**FIGURE 1:** LINC01315 may modulate miR-211-mediated DLG3 expression to participate in OSCC process. **(A)** Expression heatmap of LINC01315 in the OSCC-related expression dataset GSE30784; **(B)** Expression heatmap of LINC01315 in the OSCC-related expression dataset GSE74530; **(C)** A heatmap of differentially expressed miRNAs in the OSCC-related expression dataset GSE45238; the X axis denotes the samples, and the Y axis denotes the genes. The upper right histogram represents the color scale, where the change of color from top to bottom indicates that the expression value in the expression datasets varies in descending order. Each square depicts the expression of a gene in the corresponding sample, and each column denotes the expression of all genes in each sample. The left dendrogram denotes the clustering results among genes from different samples. The top bar denotes the sample type. The upper right box implies the level of expression, the color red indicates tumor samples, and the color blue indicates normal control samples; **(D)** Two circles respectively represent the downstream miRNAs of LINC01315 predicted using the RNA22 database and the upregulated miRNAs in the expression dataset GSE45238 and the middle part indicates the intersection miRNAs from two circles; **(E)** Expression of the miRNA candidates obtained from panel D in OSCC and normal samples in expression dataset GSE45238; the X axis refers to the miRNAs, the Y axis refers to the expression, the red box plot refers to normal samples and the blue box plot refers to OSCC samples (***p < 0.001).

### Decreased DLG3 and LINC01315 Expression but Increased miR-211 Expression in OSCC Tissues and Cells

Findings of the RT-qPCR (Figure 2A) showed that, compared with adjacent normal tissues, the OSCC tissues had higher expression of miR-211 but lower expression of LINC01315 and DLG3 (all *p* < 0.05). The results of immunohistochemistry in Figure 2B demonstrated that the positive rate of DLG3 was lower in OSCC tissues than in adjacent normal tissues (*p* < 0.05). Western blot analysis (Figure 2C) showed that the level of DLG3 protein was likewise diminished in OSCC tissues compared with adjacent normal tissues (*p* < 0.05). Moreover, Pearson correlation analysis showed negative correlations between LINC01315 and miR-211 (*p* < 0.0001, *r* = −0.5851), as well as between miR-211 and DLG3 (*p* < 0.0001, *r* = −0.5752), but a positive correlation between LINC01315 and DLG3 (*p* < 0.0001, *r* = 0.6047) (Figure 2D). Subsequently, we determined the expression of LINC01315, miR-211, and DLG3 in OSCC cells (SAS, SCC25, HN4, HN6, and CAL-27) and normal human oral keratinocytes (NHOK) by RT-qPCR. The results of this experiment revealed that, compared with NHOK cells, the SAS, SCC25, HN4, HN6, and CAL-27 cells had low expression of LINC01315 and elevated expression of miR-211 (*p* < 0.05). This difference was of highest significance in SAS and HN4 cells (Figure 2E), leading us to select these two cell lines for further experiments. Overall, our data documented that LINC01315 and DLG3 were downregulated, while miR-211 was upregulated in OSCC tissues and cells.

**FIGURE 2:** Decreased levels of DLG3 and LINC01315 but increased level of miR-211 are identified in OSCC tissues and cells. **(A)** Expression pattern of LINC01315, and miR-211 and DLG3 mRNA in OSCC tissues and adjacent normal tissues of patients with OSCC (*n* = 94) evaluated by RT-qPCR; **(B)** DLG3 positive rate in adjacent normal tissues and OSCC tissues (*n* = 94) detected by immunohistochemistry (×400); **(C)** DLG3 protein level in adjacent normal tissues and OSCC tissues (*n* = 94), as determined by western blot analysis; **(D)** Pearson correlation analysis among LINC01315, miR-211 and DLG3 expression in OSCC tissues (*n* = 94); E, Expression of LINC01315, miR-211 and DLG3 in OSCC cells (SAS, SCC25, HN4, HN6, and CAL-27) and human normal oral cell NHOK, as measured by RT-qPCR. *p < 0.05 vs. adjacent normal tissues or human normal oral cell NHOK; the data between two groups were analyzed by *t*-test and data among multiple groups were analyzed using one-way ANOVA. The experiment was repeated three times independently.

### LINC01315 Upregulates DLG3 Expression by Competitively Binding to miR-211

To investigate the relationship between DLG3 and LINC01315, we acquired base sequences of LINC01315, miR-211 and DLG3 from the NCBI database. Blast contrast analysis revealed that miR-211 had a complementary sequence both in DLG3 and LINC01315 (Figure 3A). Results of the dual-luciferase reporter gene assay (Figure 3B) revealed that the luciferase activity of LINC01315-WT in the miR-211 mimic group was attenuated compared with that in the miR-211 NC group. However, the luciferase activity of LINC01315-MUT did not differ greatly between the miR-211 mimic and miR-211 NC groups, suggesting the binding relationship between miR-211 and LINC01315. Besides, the luciferase activity of DLG3-WT-3′UTR was decreased compared with the miR-211 NC group, whereas the miR-211 mimic group did not differ from the miR-211 NC group with respect to luciferase activity of DLG3-MUT-3′-UTR (Figure 3C), further suggesting the presence of binding relationship between miR-211 and DLG3. We then performed a RIP assay to confirm further the correlations among LINC01315, miR-211, and DLG3. The results of the RIP assay showed that, compared with the IgG group, the expression of LINC01315, miR-211, and DLG3 was elevated in the argonaute 2 (Ago2) group (*p* < 0.05) (Figures 3D,E). Moreover, subcellular localization of LINC01315 was detected by FISH assay (Figure 3F), the results of which showed that LINC01315 was mainly located in the cytoplasm. The above results suggested that LINC01315 might competitively bind to miR-211 and attenuate its binding to DLG3 and indirectly regulate the expression of DLG3. To verify this speculation, we transfected SAS and HN4 cells with sh-LINC01315/sh-NC and miR-211 inhibitor/NC-inhibitor, and determined the expression of LINC01315, miR-211 and DLG3 after transfection by RT-qPCR. The results showed a reduction of DLG3 expression in OSCC cells upon LINC01315 silencing. However, DLG3 expression was upregulated in response to miR-211 inhibitor transfection. In addition, concomitant inhibition of miR-211 reversed the reduction of DLG3 provoked by LINC01315 silencing (Figure 3G). Collectively, LINC01315 could upregulate the expression of DLG3 by competitively binding to miR-211 in OSCC.

**FIGURE 3:** LINC01315 binds to miR-211 and thus upregulates DLG3 expression. **(A)** miR-211 has a complementary sequence in LINC01315 and DLG3 respectively, found by Blast contrast; **(B)** Relation between LINC01315 and miR-211 identified using dual-luciferase reporter gene assay; **(C)** Relationship between miR-211 and DLG3 identified using dual-luciferase reporter gene assay; **(D)** Binding of LINC01315 to miR-211 verified using RIP assay; **(E)**, Binding of miR-211 to DLG3 verified using RIP assay; **(F)** Subcellular location of LINC01315 determined using FISH assay. **(G)** Expression of LINC01315, miR-211 and DLG3 determined by RT-qPCR in OSCC cells transfected with sh-LINC01315/sh-NC and miR-211 inhibitor/inhibitor NC. The data were expressed as mean ± standard deviation and analyzed using one-way ANOVA. *p < 0.05 vs. the miR-211 NC group or the IgG group; ^#^*p* < 0.05 vs. the sh-NC + inhibitor NC group. The experiment was repeated three times independently.

### LINC01315 Suppresses the Proliferation, Migration, and Invasion While Inducing Apoptosis of OSCC Cells by Competitively Binding to miR-211

To explore the regulatory effects of LINC01315 on biological properties of OSCC, we assessed the proliferation, migration, and invasion abilities as well as apoptosis of SAS and HN4 cells by MTT assay (Figure 4A), scratch test (Figures 4B,C), Transwell assay (Figures 4D,E), and flow cytometry (Figures 4F,G), respectively. These analyses showed that the proliferation, migration, and invasion abilities of SAS and HN4 cells were promoted, while their cell apoptosis was attenuated in response to LINC01315 silencing. In contrast, inhibition of miR-211 attenuated proliferation, migration, and invasion abilities but enhanced apoptosis of SAS and HN4 cells. However, these cellular behaviors did not differ between the sh-LINC01315 + miR-211 inhibitor and the sh-NC + inhibitor NC groups. Altogether, LINC01315 impeded OSCC cell proliferation, migration, and invasion while stimulating cell apoptosis by binding to miR-211.

**FIGURE 4:** LINC01315 binds to miR-211 to hinder the progression of OSCC. SAS and HN6 cells were transfected with sh-LINC01315/sh-NC and miR-211 inhibitor/inhibitor NC. **(A)** Cell viability in SAS and HN6 cells assessed by MTT assay; **(B)** SAS cell migration ability measured using scratch test; **(C)** HN6 cell migration ability measured using scratch test; **(D)** SAS cell invasion ability evaluated using the Transwell assay; **(E)** HN6 cell invasion ability evaluated using the Transwell assay; **(F)** SAS cell apoptosis assessed by flow cytometry. **(G)** HN6 cell apoptosis assessed by flow cytometry. The data were expressed as mean ± standard deviation and data among multiple groups were analyzed using one-way ANOVA. *p < 0.05 vs. the sh-NC + inhibitor NC group. The experiment was repeated three times independently.

### DLG3 Activates the Hippo Signaling Pathway to Attenuate the Malignant Potentials of OSCC Cells

The above results demonstrated that LINC01315 could competitively bind to miR-211 to further elevate the expression of DLG3 in OSCC cells. Therefore, we subsequently investigated the role of DLG3 in OSCC biological functions by treating the SAS and HN4 cells with combined sh-NC and inhibitor NC, combined sh-DLG3 and inhibitor NC, and combined sh-DLG3 and miR-211 inhibitor. As determined by RT-qPCR, DLG3 expression was reduced in the sh-DLG3 + inhibitor NC group versus the sh-NC + inhibitor NC group. However, the expression of DLG3 was elevated in the sh-DLG3 + miR-211 inhibitor group as compared to the sh-DLG3 + inhibitor NC group (Figure 5A). The results of MTT assay, scratch test, Transwell assay, and flow cytometry further showed that DLG3 knockdown potentiated cell proliferation, migration, and invasion but attenuated apoptosis, whereas restoration of DLG3 by miR-211 inhibitor could reverse those effects (Figures 5B–H).

**FIGURE 5:** DLG3 silencing promotes the progression of OSCC *in vitro via* activation of the Hippo pathway. SAS and HN6 cells were transfected with sh-DLG3/sh-NC and miR-211 inhibitor/inhibitor NC. **(A)** DLG3 levels in SAS and HN6 cells after transfection detected using RT-qPCR; **(B)** Proliferation of SAS and HN4 cells after transfection measured by MTT assay; **(C)** Migration of SAS cells after transfection assessed by the scratch test; **(D)** Migration of HN4 cells after transfection assessed by the scratch test; **(E)** Invasion of SAS cells after transfection, as measured by the Transwell assay; **(F)** Invasion of HN4 cells after transfection, as measured by the Transwell assay; **(G)** SAS cell apoptosis evaluated by flow cytometry; **(H)** HN4 cell apoptosis evaluated by flow cytometry; **(I)** Expression of DLG3, MST1, MST2, LATS1 and YAP proteins in SAS cells after transfection measured by western blot analysis; **(J)** Expression of DLG3, MST1, MST2, LATS1 and YAP proteins in HN4 cells after transfection measured by western blot analysis; **(K)** Expression of YAP protein in the cytoplasm and nucleus of SAS and HN4 cells after transfection measured by immunofluorescence; *p < 0.05 vs. the sh-NC + inhibitor NC group; the data from two groups were analyzed using one-way ANOVA and the data among multiple groups at different time points were tested using repeated measures ANOVA; the experiment was repeated three times independently.

The Hippo signaling pathway mainly functions to limit the growth of adult tissues and regulate cell proliferation, differentiation and migration in developing organs. Furthermore, dysregulation of this pathway can lead to abnormal cell growth and tumorigenesis (25). LncRNA LEF1-AS1 has been reported to inhibit the progression of OSCC through the Hippo signaling pathway (20). In addition, a previous research has linked phosphorylation of YAP, a transcriptional co-activator of the Hippo pathway, to cisplatin resistance in OSCC patients (18). Based on the changes of cell function in the above experiments, we intended to examine whether Hippo pathway is involved in this process.

Next, to further detect whether DLG3 could participate in the biological processes of OSCC cells by activating the Hippo signaling pathway, we carried out western blot analysis to measure the protein levels of DLG3 and the Hippo signaling pathway-related molecules (MST1, MST2 and LATS1, and YAP). The results displayed that DLG3 knockdown resulted in downregulated levels of MST1, MST2, and LATS1 but provoked an upregulated level of YAP, whereas upregulation of MST1, MST2, and LATS1 and downregulation of YAP were seen in response to inhibition of miR-211 (Figures 5I,J). Restoration of DLG3 by miR-211 inhibitor negated the alternations in the aforementioned Hippo signaling pathway-related molecules affected by sh-DLG3. Furthermore, the immunofluorescence assay of nuclear translocation of YAP (Figure 5K) showed an increase of nuclear YAP protein after DLG3 silencing. However, miR-211 inhibitor reversed the translocation of YAP protein into nuclei induced by sh-DLG3. The aforementioned results illustrated that DLG3 silencing led to enhanced OSCC cell proliferation, migration and invasion. What’s more, DLG3 silencing increased YAP protein translocation into nuclei and slowed the apoptosis of OSCC cells.

### LINC01315 Elevates miR-211-Dependent DLG3 to Inhibit OSCC Tumor Growth in Nude Mice

To elucidate the mechanism of the LINC01315/miR-211/DLG3 axis in regulating tumor growth *in vivo*, we constructed cell lines stably co-transfected with sh-NC and inhibitor NC, sh-LINC01315 and inhibitor NC, sh-LINC01315 and miR-211 inhibitor, sh-DLG3 and inhibitor NC, as well as sh-DLG3 and miR-211 inhibitor. The results of RT-qPCR suggested that DLG3 expression was reduced, while miR-211 expression was elevated in the sh-LINC01315 + inhibitor NC group relative to the sh-NC + inhibitor NC group. However, the sh-LINC01315 + miR-211 inhibitor group exhibited an upregulation of miR-211 but a downregulation of DLG3 as compared to the sh-LINC01315 + inhibitor NC group. Moreover, miR-211 expression was unaltered, whereas DLG3 expression exhibited a downregulation in the sh-DLG3 + inhibitor NC group relative to the sh-NC + inhibitor NC group. Additionally, a reduction of miR-211 expression and an elevation of DLG3 expression were noted in the sh-NC + miR-211 inhibitor group versus the sh-NC + inhibitor NC group, and those same changes were also observed in the sh-DLG3 + miR-211 inhibitor group when compared with the sh-DLG3 + inhibitor NC group (Figure 6A). Next, these stably transfected cells were inoculated into the nude mice. The weight and volume of the tumors were measured at intervals, which showed that, compared with the mice in the sh-NC + inhibitor NC group, mice in the sh-LINC01315 + inhibitor NC group and the sh-DLG3 + inhibitor NC group had higher tumor weight and greater tumor volume, while the mice in the sh-NC + miR-211 inhibitor group had lower tumor weight and smaller tumor volume (*p* < 0.05). Corresponding tumor weights and volumes did not differ significantly among the sh-NC + inhibitor NC, sh-LINC01315 + miR-211 inhibitor, and sh-DLG3 + miR-211 inhibitor groups (Figures 6B–D). These results demonstrated that LINC01315 reduced miR-211 to upregulate DLG3, thus hindering the growth of OSCC xenograft tumors.

**FIGURE 6:** LINC01315 binds to miR-211 to increase the expression of DLG3 to further suppress xenograft tumor growth. **(A)** Expression of LINC01315, miR-211 and DLG3B determined by RT-qPCR in SAS cells transfected with sh-NC, inhibitor NC, sh-LINC01315, miR-211 inhibitor, and sh-DLG3 in combination. Nude mice were injected with SAS cells stably transfected with sh-NC, inhibitor NC, sh-LINC01315, miR-211 inhibitor, and sh-DLG3 in combination. **(B)** Representative images showing xenografts in nude mice; **(C)** Weight of xenograft tumors; **(D)** Volume of xenograft tumors measured every 1 week in nude mice; *p < 0.05 vs. the sh-NC + inhibitor NC group; ^#^*p* < 0.05 vs. the sh-LINC01315 + inhibitor NC group or the sh-DLG3 + inhibitor NC group. The data were expressed as mean ± standard deviation and analyzed by one-way ANOVA. The tumor weight and volume were measured three times independently.

## Discussion

There is an ever-increasing body of evidence that lncRNAs, like miRNAs, are differentially expressed in primary tumors and metastases (8). Furthermore, Feng et al. have confirmed that LINC01315 is differentially expressed in OSCC (6), but the detailed mechanisms by which LINC01315 functions in OSCC remain poorly understood. Therefore, we explored in this study the mechanism underlying the effects of LINC01315 on the development of OSCC, and uncovered that that LINC01315 could potentially suppress the growth of OSCC cells *via* disrupting the miR-211-mediated DLG3 downregulation.

We found that LINC01315 expression was decreased, while miR-211 expression was increased, in OSCC tissues and cells, and that LINC01315 could competitively bind to miR-211, and hence restrained SAS cell proliferation, invasion and migration, but induced cell apoptosis. This result is supported by a previous study also showing abnormal LINC01315 expression in OSCC (6). Moreover, another study has highlighted that LINC01315 is co-expressed with FAS (26), which is downregulated in OSCC (27). According to previous results, miR-211 is strongly expressed in several malignancies, such as gastric cancer, lung cancer, and OSCC (12, 28, 29), and miR-211 also acts as an oncogenic miRNA in cancer (28), as shown by the findings of Chen et al. for the case of OSCC (12). Ye et al. likewise provide evidence that miR-211 can facilitate head and neck cancer cell proliferation and invasion (11). In addition, forced high expression of miR-211 was found to enhance the proliferation, migration, and invasion of OSCC cells (5). Recent research shows that lncRNAs can function as a competing endogenous RNA to bind with miRNAs (30), and we demonstrated in this study that LINC01315 could indeed bind to miR-211, by which LINC01315 functioned to suppress progression of OSCC *in vitro*. Similarly, lncRNA maternally expressed gene 3 (MEG3) impedes the proliferation and migration of OSCC cells by selectively binding to miR-21 (31). A growing body of evidence suggests that lncRNAs can act as a competitive endogenous RNA (ceRNA) of miRNA, thus reducing their regulatory effects on mRNAs (32, 33). Here, the present findings uncovered that LINC01315 could upregulate the expression of DLG3 by competitively binding to miR-211 in OSCC. Others have also revealed a regulatory network of lncRNAs-miRNAs-mRNAs in OSCC, providing an abundance of potential therapeutic targets (34).

Additionally, we found decreased protein levels of DLG3 in OSCC tissues, suggesting that low expression of DLG3 may favor OSCC progression. When DLG3 was suppressed by shRNA, OSCC cell proliferation and invasion, and migration were promoted, but cell apoptosis was inhibited, suggesting DLG3 to be a tumor suppressor in OSCC. The DLG3 protein is a member of the membrane associated guanylate kinases (MAGUK) family (35), which are proven to be tumor suppressors (36). Indeed, a previous study has shown that DLG suppresses the growth of hematopoietic cancer (37). Our cell and animal experiments have both provided evidence supporting the conclusion that LINC01315 upregulated DLG3 expression by competitively binding to miR-211, thereby impairing the malignant phenotypes of OSCC cells.

Furthermore, we found decreased MST1, MST2 and LATS1 protein levels, and increased YAP protein levels in the nucleus of OSCC cells after downregulation of DLG3. These results demonstrate that the effects of DLG3 in OSCC are obtained *via* the Hippo signaling pathway. Recent data suggested that DLG3 is capable of binding to MST2 and then regulating LAST1, thus reducing translocation of YAP protein into nuclei (16). Furthermore, another study has revealed increased cell proliferation and decreased cell apoptosis when the Hippo signaling pathway is inactivated (38). In addition, the blocked Hippo signaling pathway is closely related to the translocation of YAP protein into the nucleus (39). Activation of Hippo signaling pathway inhibits OSCC cell survival, proliferation and migration, while enhancing cell apoptosis *in vitro* as well as arresting tumor growth *in vivo* (20), which is consistent with our present findings. Therefore, we conclude that the tumor-suppressive effect of DLG3 on OSCC cells was achieved through activation of Hippo signaling pathway.

## Conclusion

In summary, the key findings from this study demonstrated that LINC01315 could upregulate the expression of DLG3 by competitively binding to miR-211, thereby activating the Hippo signaling pathway, and inhibiting the malignant biological activities of OSCC cells (Figure 7). The results obtained from these experiments draw attention to LINC01315 as a potential target for the treatment of OSCC. However, more experiments shall be required to confirm these findings and to transform them into a practical therapy. Moreover, we suppose that the Hippo signaling pathway is not the only relevant factor in OSCC tumorigenesis which will be an interesting topic in our future researches.

**FIGURE 7:** Diagram illustrating the molecular mechanism of LINC01315 in proliferation, invasion, and migration of OSCC cells. LINC01315 can competitively bind to miR-211 and attenuate the binding of miR-211 to DLG3, which promotes the binding of DLG3 to MST1/2, leading to activation of the Hippo signaling pathway. The reduced translocation of YAP protein into nuclei correspondingly led to suppression of the proliferation, migration and invasion of OSCC cells and promotion of cell apoptosis.

## Data Availability Statement

The raw data supporting the conclusions of this article will be made available by the authors, without undue reservation.

## Ethics Statement

The animal study was approved by the Animal Committee of Ninth People’s Hospital, Shanghai Jiao Tong University School of Medicine. The human study was approved by the Ethics Committee of Ninth People’s Hospital, Shanghai Jiao Tong University School of Medicine. All subjects gave written informed consent to participate in the study.

## Author Contributions

S-CQ and XY designed the study. F-BC, XY, PW, and RZ collected clinical samples and performed the *in vitro* and *in vivo* assays. Q-XY, XZ, and R-RW analyzed and interpreted the data, and performed statistical analysis. F-BC, S-CQ, and XY reviewed the manuscript, figures, and table. All authors contributed to the article and approved the submitted version.

## Conflict of Interest

The authors declare that the research was conducted in the absence of any commercial or financial relationships that could be construed as a potential conflict of interest.

## Footnotes

1 http://www.ncbi.nlm.nih.gov/geo

2 https://cm.jefferson.edu/rna22

3 http://34.236.212.39/microrna/getMirnaForm.do

4 http://lncatlas.crg.eu/
